The article "Electroactive peptide-based supramolecular polymers" was retracted in 2022. Reason: plagiarism.

# Electroactive peptide-based supramolecular polymers

**DOI:** 10.1016/j.mtbio.2021.100099

**Published:** 2021-02-11

**Authors:** Ruslan Garifullin, Mustafa O. Guler

**Affiliations:** a Institute of Fundamental Medicine and Biology, Kazan Federal University, 420021 Kazan, Russian Federation; b The Pritzker School of Molecular Engineering, The University of Chicago, Chicago, IL, 60637, USA

**Keywords:** Self-assembly, Nanostructures, Electroactivity, Peptide-π system conjugates, Bioelectronics, Biomaterials

## Abstract

The electroactivity as a supramolecular feature of intelligently designed self-assembled systems stimulates a wide interest in development of new stimuli-responsive biomaterials. A diverse set of nanostructures are fabricated through programmed self-assembly of molecules for functional materials. Electroactive groups are conjugated as a functional moiety for organic semiconductor applications. In this review, we present recent examples of self-assembling peptide molecules and electroactive units for supramolecular functional electronic ​and optical materials with potential biomedical and bioelectronics applications.

## Introduction

There is a myriad of self-assembling molecules that already possess native electroactivity or can be conjugated with electroactive moieties. Among them, self-assembling peptides functionalized with electroactive groups present a promising future for the design of new soft materials. The self-assembly of supramolecular polymers with novel electrical and optoelectronic properties has shown significant potential in the creation of biocompatible organic semiconductors with applications in regenerative medicine and bioelectronics. The diversity of peptide functional groups in addition to the electroactive molecules enables the fabrication of multifunctional supramolecular systems. A variety of electroactive functional groups such as oligothiophene, oligopyrrole, oligoaniline, benzothienabenzothiophene (BTBT), oligophenyl, phenylenevinylene, perylene diimide (PDI), naphthalene diimide (NDI), polydiacetylene, etc. are used to fabricate supramolecular systems for bioorganic electronics ​[1].

Organic electrically conductive polymers are also used in regenerative medicine, bioelectronics, and optoelectronics. Electrically conductive polymers such as polythiophene, polypyrrole, and polyaniline have been used to promote the growth, survival, and differentiation of neural cells ​[2]. The main disadvantages of these polymers in biological applications are the problems of poor biodegradability, low water solubility, poor workability, and flexibility ​[2,3]. Preparation of composites or copolymers of these polymers with biocompatible polymers or by immobilizing peptide sequences inducing cell adhesion on the polymer chain make these polymers and their analogs more convenient for use in tissue engineering applications ​[4]. As an alternative, oligomers also provide the opportunity to develop and produce discrete and well-characterized materials with specific functionalities and properties due to their excellent solubility in common solvents and easier control over their chemical structure.

The article "Electroactive peptide-based supramolecular polymers" was retracted in 2022. Reason: plagiarism.

In this review, we present supramolecular self-assembled nanostructures as a stimulating way of construction of electroactive materials. The organization of molecules into nanostructures with ordered conductive elements provides the opportunity to obtain materials with more efficient electrical conductivity. Integration of electroactive moieties into self-assembling molecules is a promising and practical approach for potential applications in electroactive biomaterials and organic electronics. Electroactivity is closely related with molecular design and mostly depends on intramolecular π-bond conjugation; the overlapping π-orbitals create a system of delocalized π-electrons, which can give rise to outstanding optical and electronic properties. Many self-assembling π-conjugate systems utilize chromophores with semiconducting or unique photophysical properties. Supramolecular chemistry of self-assembling molecules with all its enormous richness and potential provides a basis for the rational design of hierarchical self-assembled electroactive materials. Noncovalent intermolecular interactions such as H-bonding and π-π stacking were effectively exploited to achieve self-assembly of a variety of conjugates making electron delocalization between the π-staked units possible. Several designs of self-assembling π-electron conjugates have been realized. Aromatic peptide amphiphiles (PAs), bolaamphiphiles with peptide-π-peptide units, reversed bolaamphiphiles with π-peptide-π units and peptides with π-groups as side chains are reported ​[[5], [6], [7], [8]]. This plethora of designs gives rise to various nanostructures with distinct morphologies and functions, which are the main subject of this review.

### Oligothiophene conjugates

Polythiophenes represent an important class of semiconducting materials with an example of poly (3-hexylthiophene) (P3HT), which is widely used in organic electronic devices such as solar cells and field-effect transistors (FETs). Electroactive self-assembling dendron rod coil (DRC) molecules with quaterthiophene rod segments were previously reported ​[9]. The assembly of these amphiphilic molecules into one-dimensional nanostructures is a route to π-π stacked supramolecular polymers for the development of organic materials with electronic functions. In the oligo (thiophene) DRC, self-assembly was observed to lead to three orders of magnitude increase in the conductivity of iodine-doped films. Bäuerle and coworkers were first to report a peptide–oligothiophene conjugate based on quater (3-hexylthiophene) attached to silk-inspired Gly-Ala-Gly-Ala-Gly oligopeptide sequence; optical and electrochemical properties of the conjugate were shown to be similar to those of the parent quaterthiophene ​[10]. Building on this, the polyethylene oxide (PEO) derivative of peptide-oligothiophene with enhanced solubility was synthesized ​[11]. Owing to alternating valine and threonine residues characterized by high β-sheet propensities, self-assembled fibrillar structures were observed in dichloromethane and methanol mixtures.

The article "Electroactive peptide-based supramolecular polymers" was retracted in 2022. Reason: plagiarism.

The terthiophene-conjugated tripeptide amphiphiles were shown to form helical nanofibers ​[12]. The same group also reported bolaamphiphiles based on quinquethiophene flanked by β-sheet forming tetrapeptide on both sides. In this triblock design, the addition of 6-aminohexanoic acid as a spacer was necessary to allow both π-π stacking and β-sheet formation to coexist. Microscopy revealed the formation of one-dimensional nanostructures with conductive pathways ​[13].

An electrochromic system based on a self-assembled dipeptide-flanked redox-active quinquethiophene nanofiber hydrogel is reported by the Das group (Fig. 1). The designed peptide-quinquethiophene conjugate is a symmetric bolaamphiphile that has two segments: a redox-active π-conjugated quinquethiophene core for electrochromism ​and peptide motif (Leu-Leu) for the involvement of hydrogen bonding in molecular self-assembly (Fig. 1a). The study revealed that the self-assembly and electrochromic properties of the hydrogel strongly depend on the relative orientation of peptidic and quinquethiophene structural units in the self-assembled system. The colors of the π-gel films were shown to be very stable with fast and controlled switching speed at room temperature (Fig. 1b) ​[14]. Frauenrath group used quaterthiophene–peptide conjugates to construct symmetrical multidomain structures with terminal poly (isobutylene) units. The oligopeptide-substitute quaterthiophenes self-assembled into well-ordered nanofibrils. The individual nanofibers were studied by spectroscopic and imaging methods, and the preparation of hierarchically structured microfibers of aligned nanofibrils allowed for a comprehensive structural characterization on all length scales with molecular-level precision. Thus, the molecular chirality resulted in supramolecular helicity, which supposedly suppressed lateral aggregation. Individual nanofibers comprised a single stack of the π-conjugated molecules at the core. Moreover, the conformational plasticity between the hydrogen-bonded oligopeptides and the π-π stacked chromophores produced stronger π-π interactions and hydrogen bonds. Stronger π-π stacking within the nanofibers, irrespective of the electronic features of the employed chromophores, makes them proper scaffolds to demonstrate one-dimensional charge transport along π-stacks of p-type or n-type semiconductors ​[15].

The article "Electroactive peptide-based supramolecular polymers" was retracted in 2022. Reason: plagiarism.

**Fig. 1:** a) The self-assembly of peptide-quinquethiophene-peptide bolaamphiphile into nanofiber hydrogel (π-gel), b) reversible color change of π-gel coated on ITO glass plate at operating voltage (50 ​mVs^−1^) of 0.6 ​V (yellow color) and 1.21 ​V (colorless). Adapted with permission from reference [14].

A series of peptide-oligothiophene-peptide bolaamphiphiles self-assembling in water were reported, ranging from bithiophene to sexithiophene they exhibited pH-triggered self-assembly under acidic conditions ​[[16], [17], [18]]. Moreover, torsional impacts on photophysical properties of quaterthiophene unit confined within homo-assemblies of tripeptide-π-tripeptide and its coassemblies with tripeptide-alkyl-tripeptide were discussed. The co-assembly outcome of peptide−π–peptide and peptide–alkyl–peptide conjugates into 1D nanostructures in acidic aqueous media depended on the peptide sequence and the torsional constraints imposed within the nanomaterial. In the matrix of aliphatic peptides a hydrophilic sequence Asp−Asp−Asp promoted isolation of minority π-electron components, whereas β-sheet promoting sequence Asp−Val−Val led to their clustering. Torsional restrictions exerted on the π-unit by the self-assembly process were studied on π-units with inherently different geometries, relatively planar quaterthiophene and its distorted dimethyl-substituted variant accommodating twisted bithiophene unit at the core. Deplanarization in dimethylated quaterthiophene units was shown to impede the effective π-stacking of the 1D nanoassemblies and thus modulate their photophysical properties through electronic perturbations leading to weaker exciton coupling ​[19].

Sexithiophene as a side group attached to α-helical poly (l-lysine) was reported by Holmes. This homopolypeptide self-assembled into higher order nanostructures and formed organogels in cyclohexane. The developed semiconducting material was implemented in the fabrication of organic photovoltaics and field-effect transistors ​[20].

Wan and coworkers also reported assembly of peptide–oligothiophene conjugates with two alternative designs; peptide-quaterthiophene-peptide and quaterthiophene-peptide- quaterthiophene; the conjugates were shown to form organogels in various organic solvents ​[21]. The self-assembly properties of the conjugate with the former design were also studied in solvent mixtures; nanostructures with fiber, vesicle, and parallelogram sheet morphologies were reported ​[22]. Wennemers et al. reported oligoproline-quaterthiophene conjugates with varying backbone length. Oligoprolines did not self-assemble on their own ​but controlled the organization of quaterthiophene moiety. By varying the residue number in oligoproline, a substantial change in the molecular organization of the conjugates from monolayers to double-layered sheets and helically twisted ribbons was achieved ​[23].

The article "Electroactive peptide-based supramolecular polymers" was retracted in 2022. Reason: plagiarism.

### Oligoaniline, oligophenyl, phenylenevinylene, and related conjugates

The first examples of incorporation of an extended π-electron system within an oligopeptide backbone were reported by Chmielewski and Gogoll groups; cyclic peptides with an internal azobenzene and stilbene amino acids as a conformational photoswitch were demonstrated, respectively ​[24,25]. The cis-trans photoisomerization of a conformational switch provided control over the extent of a β-turn conformation adopted by the peptides. Zhang’s group reported self-assembling aromatic peptide amphiphiles based on peptide-azobenzene conjugates. Cis-trans isomerization of the photoswitch was able to promote or impair π-π stacking of azobenzene units and intermolecular β-sheet formation, thus affecting the sol-gel transition of hydrogelator molecules (Fig. 2) ​[26]. The self-assembling peptide-π-peptide bolaamphiphile hydrogelators with biphenyl, terphenyl, and alternating thiophene-phenyl units as the central core were also shown ​[17,18].

**Fig. 2:** Cis-trans photoisomerization of peptide-azobenzene conjugate and related sol-gel transition. Adapted with permission from reference [26].

Oligo (*p*-phenylenevinylene)s (OPVs) are another well-studied class of organic semiconductors with notable fluorescence properties. One of the pioneering examples of peptide-OPV conjugates involved multiple l-lysine segments attached to a dendritic OPV unit that self-assembled in water ​[27]. Thin films prepared from the peptide-OPV conjugates were used as a surface for 3T3 fibroblasts adhesion, and the fluorescent amphiphiles were gradually internalized by the cell and accumulated in the lysosomes. Schenning and coworkers reported peptide-OPV hybrid amphiphiles that formed aggregates in organic solvents and self-assembled nanofibers in water. The amphiliphiles are composed of a oligo(p-phenylenevinylene) trimer attached to either a GAGAG silk-inspired β-sheet or a GANPNAAG β-turn forming sequence ​[28]. Building on this concept, a peptide-OPV-peptide bolaamphiphile was developed, and it self-assembles into one-dimensional nanostructures in the water at acidic pH. The design exploited carboxylic acid side chains (aspartic and glutamic acids) allowing for negatively charged and soluble peptides at neutral or basic pH [17]. Later, Mba et al. reported closely related structures forming gels in acidic and basic media ​[29]. In addition, photophysical properties were characterized, and rational approaches were developed for tuning the properties of sequence-varied peptide-OPV systems ​[30,31].

The article "Electroactive peptide-based supramolecular polymers" was retracted in 2022. Reason: plagiarism.

Oligoanilines are a class of organic semiconductors that have attracted growing interest in recent years owing to their unique redox properties and relatively high conductivity ​[32], good solubility and excellent processability ​[33], and potential use in many applications ​[[34], [35], [36], [37]]. Moreover, they produce precise chemical structures and provide opportunities for modifications and design of oligoaniline-based organic semiconductors with defined architectures, functionalities, and properties. Specifically, phenyl/amine-capped tetraaniline (TANI), a short oligomer representing the emeraldine oxidation state, is similar to polyaniline ​[32]. Our group reported a synthesis of oppositely charged aromatic peptide amphiphiles with electroactive tetraaniline in its tail part (Fig. 3). The self-assembled hydrogel of the PAs was used for neural differentiation of PC-12 ​cells; improvement in neurite outgrowth was observed on the electroactive nanofiber hydrogel with the reported conductivity of 6.97 ​× ​10^−6^ ​S ​cm^−1^ ​[38]. Schmidt’s group prepared electroactive supramolecular polymers based on oligoalanine-oligoaniline-oligoalanine conjugates. Films of the supramolecular polymer promoted adhesion of fibroblasts and provided electrically triggered release of the clinically relevant anti-inflammatory drug dexamethasone phosphate ​[39].

**Fig. 3:** Coassembly of two oppositely charged peptide-tetraaniline conjugates into electroactive nanofiber hydrogel. Adapted with permission from reference [38].

### Rylene imide conjugates

Aromatic diimides and monoimides such as perylene diimide (PDI), naphthalene diimide (NDI), and perylene monoimide (PMI) are n-type organic semiconductors, which are potential electron acceptors for solar energy conversion and molecular electronics ​[40]. Previously, bichromophoric systems exploited PDI as one of the building blocks.

Martín’s group reported an ordered donor/acceptor functional material, which has been produced by using the electrostatic coassembly method (Fig. 4). Initially, an electron-donor π-extended tetrathiafulvalene (exTTF) and an electron-acceptor PDI were separately self-assembled into n-nanofibers and *p*-nanofibers, respectively. These complementary n-nanofibers and *p*-nanofibers with oppositely charged groups on their surface established periodic alignments between nanofibers of both types resulting in a material with alternating donor/acceptor nanodomains. Photoconductivity measurements revealed electron mobility values up to 0.8 cm^2^ V^–1^ s^–1^ for these hierarchically self-assembled heterojunction structures ​[41]. Our group reported the synthesis of NDI-conjugated peptide amphiphile able to coassemble with pyrene-conjugated peptide amphiphile and form highly uniform supramolecular n/p-nanowires (Fig. 5). Supramolecular n/p-nanowires with conductivity value of 1.65 × 10^–5^ S/cm, which is about 2400 and 10 times greater compared to individual n-type and p-type nanofibers, respectively, were demonstrated ​[42].

The article "Electroactive peptide-based supramolecular polymers" was retracted in 2022. Reason: plagiarism.

**Fig. 4:** (Left) Molecular structures with schematic nanoarchitectures of exTTF derivative and PDI derivatives. (Middle-Right) Schematic representation of the n/p-material obtained by the coassembly of previously self-assembled molecules. Adapted with permission from reference [41].

**Fig. 5:** Coassembly of p- and n-type peptide-chromophore (PC) conjugates into charge-transfer complex nanofibers. Adapted with permission from reference [42].

Bartocci et al. also reported charge-transfer organogels formed by coassembly of NDI- and pyrene-conjugated diphenylalanine. Electronic paramagnetic resonance measurements revealed the advantage of preorganized charge-transfer supramolecular architectures for charge transport ​[43].

Ghadiri group developed self-assembling cyclic D,L-α-peptides composed of alternating *D*- and *L*-residues as a template to achieve hydrogen bond-directed ring stacking and charge transfer between NDI side chains ​[44,45]. Studies of the structural and photoluminescence properties of the conjugates in solution showed that the hydrogen bond-directed assembly of the cyclic D,L-α-peptide backbone promotes intermolecular NDI excimer formation. The efficiency of NDI charge transfer in the resulting construct depends on the length of the linker between the NDI and the peptide backbone, the distal NDI substituent, and the number of NDIs attached [44]. The same peptide backbone was used for redox-promoted self-assembly of cyclic peptide with four NDIs attached; reversible reduction of the NDI side chains to the corresponding NDI anion radicals resulted in the formation of peptide nanotubes with extended charge-delocalized states [45]. Parquette et al. reported dilysine-NDI peptide amphiphiles functionalized with NDI at the ε-amino position of either of lysine residues, Ac-KK(NDI) and Ac-K(NDI)K ​[46]. Furthermore, an effect of groups with increasing hydrophobicity (H-, acetyl-, and Fmoc substituents) at the *N*-terminus of the peptide was studied. Only acetyl- and Fmoc-substituted variants assembled into 1D n-type nanostructures in water, with latter one forming hydrogel ​[47]. These NDI-appended PAs formed one-dimensional n-type nanostructures in water and forming a self-supporting hydrogel. The same group reported the self-assembly of lysine-NDI-lysine bolaamphiphile and lysine-NDI-butyl amphiphiles into nanotubular structures ​[48,49]. Ashkenasy et al. reported amphiphilic peptide with NDI moieties as side chains that assembled into fibrils with substantial intermolecular π-stacking ​[50].

The article "Electroactive peptide-based supramolecular polymers" was retracted in 2022. Reason: plagiarism.

The pH-responsive VDFAG-NDI-GAFDV and VDFAG-PDI-GAFDV conjugates assembling into one-dimensional nanostructures with H-type aggregation at acidic pH were also shown ​[17]. Hodgkiss also presented peptide-PDI-peptide bolaamphiphiles with detailed elaboration on ionic effects and solvatochromism in the aggregation of the peptide-PDI units ​[51]. The H-aggregate formation was considerably enhanced by zinc dication coordinating to two glutamate residues at neighboring molecules. The same group reported a spectroscopic investigation of assembly in an extensive series of peptide-PDI conjugates specifically designed to analyze the effect of structural variations. By fitting different contributions to temperature-dependent optical absorption spectra, the thermodynamics and the nature of peptide aggregation were quantified based on incremental variations in peptide hydrophobicity, charge density, as well as asymmetric substitution with a hexyl chain, and stereocenter inversion. The hydrophobicity and hexyl substitution were shown to have the most effect on self-assembly thermodynamics, which ais formed by enthalpic and entropic influences. Moreover, significant peptide packing effects were resolved via stereocenter inversion studies focused on the the nature of aggregates and the coupling between π orbitals. The results established a quantitative framework for deriving structure−function correlations that can outline the design principles of self-assembling peptides for electronic materials ​[52]. Frauenrath et al. reported self-assembly of peptide-PDI-peptide with terminal poly(isobutylene) units to obtain well-ordered nanofibers. The conformational flexibility between the hydrogen-bonded oligopeptide segments and the π-stacked chromophores gave rise to synergistically enhanced π-π interactions and hydrogen-bonds ​[15].

The reversible in situ formation of a self-assembling building block, NDI–dipeptide conjugate, by enzymatic condensation of NDI-functionalized tyrosine and phenylalanine-amide to form NDI-YF-NH_2_ is reported by the Ulijn group. This biocatalytic self-assembly is thermodynamically driven and produces nanostructures with improved supramolecular interactions, as shown by aggregation-induced emission. In the presence of dihydroxy/alkoxy naphthalene (DHN/DAN) donors, charge-transfer complexes are generated. These dynamic nanostructures, whose formation and function are driven by free-energy minimization, are inherently self-healing and provide opportunities for the development of adaptive nanotechnology ​[53]. The same group demonstrated amino-acid-encoded biocatalytic self-assembly that enabled the formation of transient conducting nanostructures. Amino acids were used to modify a self-assembling core unit in situ, thereby controlling its amphiphilicity and consequent mode of assembly. The core NDI unit was flanked by D- and L-tyrosine methyl esters as competing reactive sites. Kinetic competition between ester hydrolysis and amidation resulted in covalent or noncovalent amino acid incorporation in the presence of α-chymotrypsin and selected encoding amino acid. Owing to the NDI core, electronic wires formed and subsequently degraded, demonstrating a temporally regulated electronic conductance ​[54].

The article "Electroactive peptide-based supramolecular polymers" was retracted in 2022. Reason: plagiarism.

Wennemers et al. presented conjugates between oligoprolines and sterically demanding perylene monoimides (PMIs) that form hierarchical supramolecular ensembles. The effect of the backbone length, the stereochemistry at the attachment site, and the location of the chromophore on the self-assembly properties of the conjugates was studied. Self-assembled nanostructures that range from flexible worm-like threads via bundles of rigid fibers to nanosheets and nanotubes were observed ​[[55], [56], [57]]. The same group reported a triaxial supramolecular weave that consists of self-assembled organic threads; each thread is formed by the self-assembly of a building block comprising a rigid oligoproline backbone appended by two PMI chromophores. The π-stacking of the chromophores results in threads that feature alternating up and down-facing voids at regular distances. The voids accommodate incoming building blocks and establish crossing points through CH–π interactions ​[58].

### Polydiacetylene conjugates

Polydiacetylenes (PDAs) and their supramolecular structures are also of particular interest, as they possess distinct chromic and sensing properties ​[[59], [60], [61]]. PDAs exist in two distinct conformational extremes, which are a nonfluorescent blue phase and a fluorescent red phase ​[62,63]. The monomeric diacetylene (DA) undergoes topochemical polymerization via 1,4-addition ​when strict geometric requirements are met by the precursor crystal (Fig. 6) ​[64].

The article "Electroactive peptide-based supramolecular polymers" was retracted in 2022. Reason: plagiarism.

**Fig. 6:** Topochemical polymerization of DA monomers (a) and different conformations of the PDA backbone (b) showing a rigid rod form with maximum conjugation (i), a linear conjugated segment (LCS) structure with discrete breaks in conjugation (ii), continuous deformation of a backbone resulting in decreased conjugation (iii) and a highly disordered ‘coil’ with cis-double bonds (iv). Adapted with permission from reference [64].

Frauenrath et al. reported an amphiphilic system that makes use of hydrogen-bonded peptide segments to preorganize diacetylene units and promotes the polymerization within hydrogel or organogel networks. The first-generation peptide–diacetylene conjugates comprised poly (isoprene) tail providing solubility in organic solvents, tetra (L-alanine) repeat for β-sheet formation, and the polymerizable diacetylene in the head of the structure. Polymerization resulted in the formation of flat ribbon and tape-like nanostructures ​[65]. Peptide-diacetylene-peptide bolaamphiphiles with terminal L-glutamate residues were synthesized by Wang’s group; synthesized peptide–polydiacetylene conjugates with aliphatic linkers formed fiber-like nanostructures in water ​[66]. Related structures were reported by Liu and coworkers, a bolaamphiphile with diacetylene mesogen core was designed, and the compound was found to form a photopolymerizable hydrogel in water ​[67]. Tovar group also reported self-assembling peptide-π-peptide bolaamphiphiles with diphenyl butadiyne as the polymerizable unit, demonstrating reversible pH-dependent blue–red phase transition ​[68].

Liu and coworkers reported a synthesis of amphiphilic amino acid-diacetylene conjugate, where an L-glutamic acid was modified with unsaturated 10,12-Tricosadiynoic acid (Fig. 7). The conjugate was found to self-assemble into vesicles in water and supramolecular gel with helical structures in binary methanol-water solvent. The vesicles and the helices showed topochemical photopolymerization under UV irradiation and showed a blue color. After the self-assembly and photopolymerization, the chirality of localized L-glutamic acid was transferred to polydiacetylene (PDA), which was shown by circular dichroism (CD) signals in the PDA blue phase. Obtained supramolecular structures showed effective enantioselective recognition of sulfinamide enantiomers, in which the assemblies with S-enantiomer turned red while the other remained blue in the presence of the R-enantiomer ​[69]. The peptide amphiphile structures with unsaturated hydrocarbon tail, where peptide sequences were conjugated with 10,12-pentacosadiynoic acid, were reported. The PAs assembled into nanofibers that formed PDA hydrogels in the blue phase with temperature-dependent chiroptical properties ​[70]. The van Hest group reported a study of pH and temperature dependence of self-assembly of related PAs with varying alkyl tail length. It was shown that the length of the alkyl chain changed the assembly and disassembly temperatures, while pH did not have a substantial influence on the nanostructures. Polymerized, the molecular packing of the PAs was just barely influenced by temperature increase, as indicated by reversible small color change of PDA fibers ​[71]. The effect of the DA position within alkyl tail on the chromatic properties of polymerized self-assembled PA fibers was also reported [72]. They also reported a possibility to magnetically align peptide amphiphile containing diacetylene moiety in the alkyl tail and obtain polymerizable nanofibers with high order ​[73].

The article "Electroactive peptide-based supramolecular polymers" was retracted in 2022. Reason: plagiarism.

**Fig. 7:** Illustration on the formation of PDA-Glu vesicles and helices and their selective recognition of enantiomers of tert-butylsulfinamide. Adapted with permission from reference [69].

### Other π–peptide conjugates (tetrathiafulvalenes, thienyl, BTBT, Fmoc, pyrene)

We presented a class of semiconductor nanowires formed by the supramolecular assembly of amphiphilic benzothienabenzothiophene (BTBT)-peptide conjugates (Fig. 8). The electroactive BTBT unit was for the first time utilized in the preparation of self-assembled one-dimensional peptide nanostructures in aqueous media. β-sheet forming peptide amphiphiles self-assembled into highly uniform nanofibers with a diameter of c.a. 10 ​nm and micron-size lengths. We also showed the presence of the J-type π–π staking among the BTBT units throughout the hydrophobic core of the self-assembled nanofibers yielding an electrical conductivity as high as 6.0 ​× ​10^−6^ ​S ​cm^−1^ ​[74].

**Fig. 8:** Molecular structures of amphiphilic BTBT–peptide conjugates, the BTBT–peptide (BTBT–C3-COHN-Ahx-VVAGKK-Am), and the C8-BTBT–peptide (C8-BTBT–C3-COHN-Ahx-VVAGKK-Am). (b) A schematic representation of the self-assembly process for the BTBT–peptide amphiphile showing the proposed nanofiber structure with the computed molecular length (∼4.4 ​nm) and the measured nanofiber diameter (∼11 ​± ​1 ​nm). Adapted with permission from reference [74].

Non-natural thienyl alanine amino acids were used to synthesize self-assembling thienyl-containing oligopeptides. Electronic properties of β-sheet fibrils are expected because of charge delocalization and π-stacking; the formation of hydrogels in a concentration-dependent manner holds the potential for the development of responsive nanomaterials incorporating electronic functionality ​[75,76]. N. Ashkenasy group reported electron and proton mediated charge transport of self-assembled nanostructures of the peptide functionalized with thienyl moiety under low humidity conditions, and proton transport dominated conductance at higher relative humidity ​[77].

The article "Electroactive peptide-based supramolecular polymers" was retracted in 2022. Reason: plagiarism.

Thiophene-based structure such as 3,4-ethylenedioxythiophene (EDOT) was also used to obtain conducting polymers. Conducting polyEDOT (PEDOT) polymers confined within bioactive peptide amphiphile nanofibers were reported. PA, palmitoyl-AAAAGGGEIKVAV, was allowed to self-assemble from its aqueous solution in the presence of a hydrophobic EDOT monomer. The hydrophobic core of the nanofibers that form as the PA molecules self-assemble in water encapsulates EDOT monomers, whose polymerization into PEDOT is achieved by chemical or electrochemical means ​[78]. Murphy’s group reported templating the 3D structure of conducting polymers with self-assembling peptides. In the first study, peptide-EDOT conjugate, hexyl-GAGA-EDOT, was observed to assemble into fibrous networks in organic solvents, revealing a soft gel. When assembled peptide gels were exposed to in situ oxidative polymerization of the peptide-bound and free hydroxymethyl-EDOT (EDOT-OH) monomers, a network of conductive nanowires formed ​[79]. In another study, a series of tetrapeptides XYXA and XXYA, where X ​= ​L or V and Y ​= ​E or D, conjugated with 3-thiopheneacetic acid at *N*-terminus, were self-assembled into β-sheet containing gels in the presence of exogenous EDOT-OH. The gels were subjected to oxidative polymerization, and gels with conductivities approaching that of pure PEDOT and undoped silicon were obtained. All gels had similar fibrous, porous structures with β-sheet structural motif before and after polymerization ​[80].

Kato et al. reported electroactive supramolecular nanofibers assembled from oligopeptide-tetrathiafulvalene (TTF) conjugates. These nanofibers are one-dimensional hydrogen-bonded systems with electroactive groups showing electrical conductivity obtained after doping with iodine. In addition, partial oxidization of the TTF groups after exposure to iodine led to an obvious improvement in stacking and more thermally stable fibers ​[81]. Martín et al. synthesized peptides functionalized with concave 9,10-di (1,3-dithiol-2ylidene)-9,10-dihydroanthracene (exTTF) units, resulting in multilamellar supramolecular helical assemblies. An assembly of twisted flat ribbon-like structures in chloroform and methylcyclohexane was observed as a result of three-dimensional supramolecular ordering at the mesoscale due to solvophobic collapse ​[82,83]. Recently, Kimura and co-workers reported conjugates of TTF and chloranil with cyclic tripeptides that individually and in combination self-assemble into peptide nanotube (PNT) bundles. Co-assembled PNT architecture provided alignment of TTF (donor) and chloranil (acceptor) with formation of charge-transfer complexes. Surface potentials of co-assembled PNT bundles were greater compared to mixture of individual PNTs. The bundles demonstrated a hysteresis response in the piezoelectric force curve with varying bias voltages according to piezoelectric force microscope measurements [84].

The article "Electroactive peptide-based supramolecular polymers" was retracted in 2022. Reason: plagiarism.

Self-assembling peptides conjugated to fluorenyl-9-methoxycarbonyl (Fmoc) group and/or with multiple phenylalanine residues offer additional π–π interactions, which can guide supramolecular assembly, giving rise to a myriad of new π-conjugated peptides with optoelectronic activity. Many independent studies carried out by Adams, Gazit, Ulijn, and Xu groups have provided detailed information on the properties and self-assembly mechanisms of Fmoc-based and oligophenylalanine-based molecules that effectively form self-supporting gels ​[5,[85], [86], [87], [88], [89]]. The naphthalene, pyrene, diketopyrrolopyrrole, and a number of small aromatic compounds have been exploited to synthesize low molecular weight peptide gelators ​[90]. Adams group developed dipeptide-π-dipeptide bolaamphiphile with diketopyrrolopyrrole as an aromatic core. The conjugate was shown to form a hydrogel upon pH change. Not only this gelator formed entangled aggregates at low pH, but it also morphed into worm-like micelles at high pH. The structures at high pH could be further processed by using shear to form aligned structures with directional dependence and improved conductivity ​[91]. Banerjee’s group reported the self-assembly of a pyrene–peptide conjugate that resulted in a transparent self-supporting gel in organic solvents and is fluorescent in o-dichlorobenzene ​[92]. We also reported peptide amphiphile with pyrene in its tail part; the molecule assembled into nanofibers in water and formed nanofiber gel at basic pH. Helical organization and π-π stacking of pyrene units throughout nanofibers had a tremendous impact on the photophysical properties of achiral chromophore manifested in emergence of chiropticity ​[93]. Kato and coworkers reported one-dimensional chiral self-assembly of the dendritic oligopeptide-pyrene conjugate. The conjugate had a molecular triblock structural design: pyrene moieties at focal points, branched oligo (glutamic acid)s as chiral hydrogen-bond introducing parts ​and lipophilic alkyl parts. The molecule formed cylindrical columns by nano-segregation between the molecular block structures. The addition of an equimolar amount of 2,4,7-trinitrofluorenone (TNF) to the conjugate resulted in an electron donor-acceptor complex of dark red color with induced hexagonal columnar phase. The properties of the π-extended functional groups, including luminescence, electron conductivity, and ferroelectricity, can be tuned by chiral supramolecular structures composed of a number of intermolecular interactions ​[94].

The article "Electroactive peptide-based supramolecular polymers" was retracted in 2022. Reason: plagiarism.

The integration of a naphthalene-tripeptide (Phe-Phe-Lys) conjugate, which is a versatile self-assembly motif, with a redox-active ruthenium-(II)tris (bipyridine) complex was reported by Xu and coworkers (Fig. 9a). It is the first metallo-hydrogelator that self-assembles in water, forming a hydrogel, and exhibits gel−sol transition by oxidation of the metal center (Fig. 9b). The addition of the metal complex in the hydrogelator causes a self-assembly process forming nanofibers with the size of a single molecule of the hydrogelator. Therefore, the metal complexes provide optical, electronic, redox, or magnetic properties to the supramolecular hydrogels. The metal complexes were used to moderate the intermolecular interactions to elucidate the mechanism of formation of the molecular nanofibers to enable the development of functional supramolecular hydrogel materials ​[95].

**Fig. 9:** a) Molecular structure and space-filling model of the metallo-hydrogelator, b) optical images of oxidation-induced gel−sol transition and the TEM images corresponding to the samples at different states of transition. Adapted with permission from reference [95].

Larger aromatic systems such as aromatic macromolecules, carbon-rich compounds, and even carbon allotropes are also widely used in the preparation of electroactive and photoactive self-assembled functional materials. The C-terminal conjugates of α-helical polypeptide alamethicin (F30) with C_60_ or C_70_ fullerenes were reported to form self-assembled voltage-dependent ion-conducting channels. Voltage-dependent bilayer experiments revealed preferred channel sizes for F30–C_60_ and –C_70_ conjugates and higher activity compared with native alamethicin; moreover, latter conjugate exhibited pore states with remarkably long lifetimes of seconds ​[96]. Conjugates of β- and γ-diphenylalanine with carbon nanotubes (CNTs) were observed to self-assemble into fibrillar dendritic structures ​[97]. As an example of noncovalent involvement, three different oxidized nanocarbons - 1D CNT, 2D graphene oxide (GO) sheet, and 3D carbon nanohorn (CNH) - were studied for their effects on the self-assembly of the Leu-^D^Phe-^D^Phe tripeptide at physiological conditions. Viscoelastic properties of supramolecular hydrogels were clearly affected by the nanocarbons, manifested by an increase in stiffness and resistance to applied stress. Notably, hydrogel self-healing behavior was observed only with embedded CNTs. Experimental and in silico investigation of the tripeptide-CNT interaction suggested that the latter acts as a nucleation center for self-assembly and reassembly ​[98]. Hydrogels were also reported for Fmoc-Phe and oxidized CNTs ​[99], and Fmoc-Phe-Asp/Fmoc-Tyr-Asp, and reduced GO ​[100]. In all cases, the inclusion of the nanocarbons led to an increase in stiffness. Further, carbon-rich hexa-peri-hexabenzocoronenes (HBCs) are known for their π-π stacking promoted high self-assembly potential and are well-studied with the aim of further implementation in organic electronic devices. To further direct supramolecular organization processes, Gemini-shaped amphiphilic HBC derivatives carrying chiral hydrophilic substituents were constructed by Zhang and coworkers. Native HBCs and fluorine-substituted HBCs self-assembled into nanotubular structures and nontubular aggregates, respectively, which are CD-active ​[101]. A water-soluble hexa-peri-hexabenzocoronene molecule with peripheral functional groups self-assembles in water and forms fibers by π-π stacking and consequent peptide binding through electrostatic interactions. First, the HBC derivative self-assembled into water-soluble red-fluorescent fibers that served as a template for further modification with biomolecules. Then, the peripheral negatively charged functional groups bind positively charged green-fluorescent fluorescein-peptide conjugate, producing well-defined fibers that were visualized as dual-color fibers in double-fluorescence imaging ​[102]. A similar electrostatic binding strategy was used by Fairman and coworkers with an anionic porphyrin (mesotetrakis (4-sulfonatophenyl)porphyrin) that induced a coiled-coil structure in an oligopeptide via cationic lysine residues. The binding was demonstrated by the intensity decrease in the Soret band of porphyrin at 413 ​nm with increasing peptide concentration ​[103]. The inclusion of metal coordinating groups in self-assembling molecules was also exploited to organize metal-complex chromophores. Long fibers assembled from peptide amphiphiles capable of binding the metalloporphyrin zinc protoporphyrin IX have been reported. A palmitoyl-AHL_3_K_3_ peptide was synthesized for supramolecular fiber formation. A porphyrin-binding site, a single histidine, was added into the peptide structure to bind zinc protoporphyrin IX for photophysical properties. A reduced hemin ​(PPIX)Fe^II^ ​was also exploited for more tunable optical properties ​[104]. Solomon and coworkers also reported three self-assembling peptide amphiphiles that have heme-binding sites either on the hydrophobic or hydrophilic face of the peptide. They differ significantly in their morphologies and heme-binding properties. A relatively weak heme binding was observed for palmitoyl-(LK)_3_ as its binding site lay on the hydrophilic side of the peptide assembly, yielding low binding affinity. Two other PAs, palmitoyl-L_3_K_3_ and palmitoyl-(KL)_3_, yielded distinct morphologies, fibers, and sheets, respectively, but both bound heme with relatively high binding affinities. While the redox properties of the heme molecules were apparently unaffected, the electronic characterization suggested that palmitoyl-(KL)_3_ favored a slipped, cofacial arrangement of heme molecules, as shown by the split Soret band. The study demonstrates a wide spectrum of opportunities when designing peptides for different energy applications. These findings suggest that the peptides serve ​as a scaffold for material design and provide a library of tools to electronically modulate energy-relevant molecules such as heme ​[105]. Zinc phthalocyanine−peptide conjugates were synthesized by Sonogashira cross-coupling of an iodinated zinc phthalocyanine with acetylenic bombesin protein or Arg-Gly-Asp (RGD) tripeptide motif. They are used as potent photosensitizers for the imaging and photodynamic therapy of tumors ​[106]. In addition, noncovalent patterning of zinc phthalocyanine derivative in the core of self-assembled peptide amphiphile nanofibers was reported by our group; encapsulated chromophore molecules were organized via hydrophobic and Van der Waals interactions throughout the hydrophobic interior of nanofibers. Peptide nanofibers acted as a supramolecular cavitand forcing chromophore molecules to attain face to face organization (H-aggregates) and inducing fast energy transfer, which was evidenced by complete fluorescence quenching ​[107].

The article "Electroactive peptide-based supramolecular polymers" was retracted in 2022. Reason: plagiarism.

### Electrical and photophysical (optical) properties

Supramolecular organization of molecularly discrete holons into the structures with higher complexity, expectedly, unlocks supramolecular features of π-electron systems involved in self-assembled peptide ensembles and gives rise to new optoelectronic properties. Therefore, changes in absorption and emission spectra are typically used as evidence of supramolecular polymerization. Spatially unique chromophore aggregation and mutual orientation entail ​modulation of the optical response of the supramolecular material ​[[108], [109], [110]]. Wall et al. carried out studies on the effects of amino acid sequence [30,111] and formal hydrogen bonding networks [31] on optoelectronic properties of π-conjugated peptide ensembles. Variations in the amino acid sequence or formal hydrogen bonding directionality did not result in any substantial changes in the self-assembly potential of the molecules, in contrast to photophysical responses ranging from long-lived excimeric to short-lived excitonic states ​[111]. Kiick et al. also reported exciton-coupling variations stemming from variations in the distances between the π-electron units attached to α-helical peptide ​[112,113]. Along with variations in the absorption spectra, the CD spectra were also highly dependent on distance and dihedral angle between the chromophores ​[112]. We reported that supramolecular chirality and related CD spectra were induced in the pyrene chromophore by PA assembly into chiral nanostructures, whether it was covalently attached ​or noncovalently bound. The mode of interaction of β-sheet forming sequence with the chromophore in final supramolecular polymer considerably affected CD spectra ​[52]. Variation in the π-electron moiety location, peptide-π-peptide or π-peptide-π design, was also studied by Guo et al., demonstrating H-aggregation for both designs, but with tighter π–π packing for the former one ​[21]. Optical properties of the self-assembled systems are used for imaging the nanostructures in biodiagnostics and drug delivery applications. Conjugation of chromophores is also useful in measuring diffusion properties of the nanoparticles and phototherapy applications ​[114].

There are numerous reports on the inherent or induced conductivity of proteins and peptides ​[[115], [116], [117], [118]]. In this context, one of the extensively studied peptides is diphenylalanine and its derivatives ​[119]. Its ability to self-assemble into nanotubes in solution, as well as from vaporous phase, has made this dipeptide a model structure in studying various manifestations of electroactivity ​and enabled its use in device applications ​[120,121]. Gazit’s group demonstrated the self-assembly of large arrays of aromatic dipeptide nanotubes (ADNTs) from diphenylalanine precursors using the vapor deposition method. During evaporation at elevated temperatures (up to 220 ​°C), the diphenylalanine molecules (Phe-Phe) attained a cyclic structure (cyclo–Phe–Phe) and then assembled on a substrate to form ordered vertically aligned nanotubes. This method allowed control of the length and density of the nanotubes by changing the building blocks. It was also shown that the nanotube arrays provide high-surface-area electrodes for energy storage, hydrophobic self-cleaning surfaces, and microfluidic platforms. For instance, electrostatic ultracapacitors based on ADNT-modified carbon electrodes were fabricated. The ADNT arrays enabled a large functional surface area for the ultracapacitor electrodes and significantly increased their capacitance. The ADNT modified carbon electrodes are expected to enable significant growth of the electrical double-layer capacitance density, reaching C_DL_ ​= ​480 ​μF ​cm^−2^ for a geometric electrode area; in contrast, C_DL_ ​= ​16 ​μF ​cm^−2^ for the carbon electrode ​[120].

The article "Electroactive peptide-based supramolecular polymers" was retracted in 2022. Reason: plagiarism.

Rosenman and coworkers showed anomalously strong shear piezoelectric activity in self-assembled diphenylalanine nanotubes associated with electric polarization along the tube axis ​[122]. Building on that, self-assembled diphenylalanine material-based energy harvesters were demonstrated ​[[123], [124], [125]]. The peptide-based piezoelectric energy harvesters could generate a voltage, current, and power of up to 2.8 ​V, 37.4 ​nA, and 8.2 ​nW, respectively, with 42 ​N of force, powering multiple liquid crystal display panels ​[123]. Ferroelectric behavior of self-assembled diphenylalanine tubular structures was also observed due to the alignment of dipoles ​[126,127]. The difference in impedance between the electrodes enables the detection of proteins and pathogens with the contribution of ferroelectric peptides assemblies ​[128]. The electrical properties of certain π-peptide conjugates strongly correlate with the specific peptide sequence and the consequent structural motif. For instance, the investigation of bulk electrical properties of conductive films composed of peptide-oligothiophene nanostructures and its dependence on the amino acid sequence showed that the inherent aggregation into films varies simply through peptide substitutions ​and consequently affects the surface roughness of the films, which is correlated with the sheet resistance of the material ​[111]. These results are also linear with the pure peptide conductance ​[115]. Akdim et al. in silico demonstrated that π-electron-rich amino acids such as phenylalanine, tyrosine, and tryptophan in self-assembling peptides are essential for conductivity behavior ​[129]. Nevertheless, some studies suggest that the supramolecular ordering and secondary structure of building blocks of the self-assembled peptide nanostructures can be not less critical structural features in supporting electronic conductivity. Hochbaum group demonstrated long-range electronic transport in biomimetic α-helical peptide nanofibers and gels lacking the extended conjugation, π-stacking, or redox centers typical of existing organic and biohybrid semiconductors. The supramolecular structure of the peptide nanofibers precluded π orbital overlap between side chains of aromatic amino acids, suggesting a mechanism of conduction distinct from the band conduction of periodic, π-stacked organic materials. Electrochemical transport measurements revealed that the fibers support ohmic electronic transport and metallic-like temperature dependence of conductivity in an aqueous system ​[130].

The article "Electroactive peptide-based supramolecular polymers" was retracted in 2022. Reason: plagiarism.

Peptide-oligothiophene hydrogelators were used as active layers of FETs, demonstrating hole mobilities in the range of 10^−5^ – 0.03 ​cm^2^ ​V^−1^ s^−1^ ​[18,131]. The observed values are higher than that of hairpin-shaped sexithiophene ensembles (μh ​≈ ​10^−7^–10^−6^ ​cm^2^ ​V^−1^ s^−1^) with amide hydrogen-bonding or the OFET devices with α-helical peptide-based oligothiophenes as the semiconductor (μh ​≈ ​10^−8^–10^−7^ ​cm^2^ ​V^−1^ s^−1^) ​[20,132]. Electrostatic force microscopy was used to qualitatively assess the potential of peptide–polydiacetylene conjugates in facilitating the movement of charge carriers, demonstrating a new approach to the analysis of electrical conductivity with no physical electrode deposition required ​[68,133]. A layer-by-layer deposition methodology of Tyr/Trp-containing short self-assembling cyclic peptides, which results in vertically oriented nanotubes on gold substrates, was reported by N. Ashkenasy group. By using this novel deposition methodology, molecular junctions with a conductive atomic force microscopy tip as a second electrode were fabricated. Studies of the junction current–voltage characteristics as a function of the nanotube length revealed an efficient charge transfer in these supramolecular structures, with a low current attenuation constant of 0.1 ​Å^−1^, which indicated that electron transfer is dominated by hopping. The threshold voltage to field-emission dominated transport was found to increase with peptide length in a manner that depends on the nature of the contact with the electrodes. Tailorable peptide molecules and their self-assembled nanostructures are potentially important for engineering electroactive self-assembled peptide nanotubes for bioelectronics applications ​[134].

### Biomedical applications of electroactive materials

Electroactive supramolecular polymers are of great interest to the medical field due to their electrical/optical properties and potential tissue compatibility. Conventional conductive polymers alone are hard to process into useful three-dimensional architectures due to their intrinsic brittleness, which limits their use to thin coatings. Therefore, the development of easily processable biocompatible electroactive materials is necessary to extend the practical use of supramolecular polymers into bio-stimulation, neural recording/modulation, artificial tissue engineering, and drug delivery. By engineering biocompatible self-assembled materials based on peptide-π system conjugates with tunable properties and physical morphology, the use of supramolecular polymers for fields such as neuroscience and prosthetics can be achieved. In recent years, self-assembling peptides have been employed to organize small molecule semiconductors ​[7]. Self-assembly is useful for achieving large-scale, tunable organization with anisotropic conductivity. Oligomer systems demonstrated conductivities, which are limited to the semiconducting range, making it difficult to interface these materials with the electronics required for bio-stimulation applications. The use of peptides to organize monomers for in situ polymerization and preparation of highly conductive polymers would enable more efficient device fabrication. Thus far, only a limited number of studies have implemented the aforementioned strategy to form polydiacetylene [68,71,135] or PEDOT [78] nanowires insulated by the bioactive shell with the best-reported conductivities on the order of 10^−5^ ​S ​cm^−1^. As potential applications of electroactive supramolecular polymers encompass neural stimulation electrodes, drug delivery systems, artificial muscles, nerve conduits, and engineered tissue scaffolds, matrices with biologically relevant mechanical properties and architectures are required. Porous electroactive hydrogels with conductivities c.a. 10^−2^ ​S ​cm^−1^ and moduli range of 20–120 ​kPa, which fall in the same range as breast (2–20 ​kPa), brain (30–100 ​kPa), and heart tissues (10–5000 ​kPa), are made available through additional covalent polymerization of electroactive thiophene-based units ​[80].

The article "Electroactive peptide-based supramolecular polymers" was retracted in 2022. Reason: plagiarism.

Preliminary in vivo experiments showed that supramolecular systems of peptide-π system conjugates hold a promising therapeutic potential and can be implemented in various biomedical applications. Coexistence with biologically relevant fragments such as peptide sequences should ameliorate the toxicity profile of π-conjugated systems and provide reasonable clearance. Nevertheless, biological aspects such as cytotoxicity and genotoxicity should be thoroughly studied. The electrical conductivity of hydrogels is crucial for their applications with cardiac, skeletal, and neural cells, which exhibit electroactive dependence behavior ​[2]. So far, electroactive supramolecular polymers have been used as both biologically and electronically active scaffolds for the transduction of biological events such as cell stimulation and intercellular communication. Self-assembled PA hydrogel with electroactive tetraaniline unit was used for neural differentiation of PC-12 ​cells with improvement in neurite outgrowth [38]. Supramolecular polymer films of peptide-oligoaniline conjugate promoted adhesion of fibroblasts and provided electrically triggered release of the anti-inflammatory drug ​[39]. Thin films of peptide-OPV conjugates were used to promote 3T3 fibroblasts adhesion; however, an analogous pyrene-based conjugate was cytotoxic ​[27]. Fmoc-diphenylalanine peptides have also found applications in drug delivery ​[136], biological sensing [137], and cell culture [[138], [139], [140], [141]] owing to their ability to assemble into nanofibers and form hydrogels under physiological conditions; however, Fmoc and pyrene are reportedly carcinogenic, and therefore, other alternatives such as naphthalene moiety, which is a common fragment of many clinically approved drugs, should be considered ​[100]. Peptide–naphthalene conjugates have high gelation efficiencies (as low as 0.07 ​wt %), demonstrate reasonable cytological compatibility ​[100,142], and even can be rendered proteolytically stable with the inclusion of d-amino acids ​[143]. A series of glycosylated aromatic peptide amphiphiles based on naphthalene-FFDD conjugate exhibited diverse self-assembling behaviors in water and formed supramolecular hydrogels with enhanced thermostability and biostability compared to their parent conjugate ​[144].

The article "Electroactive peptide-based supramolecular polymers" was retracted in 2022. Reason: plagiarism.

Dendritic supramolecular assemblies of β-homologated and γ-homologated diphenylalanines conjugated with CNT enabled the growth of primary hippocampal cells and the modulation of their neuronal functions. The geometrical restrictions imposed by CNT nucleated nodes allowed the growth of neuronal networks with control over network geometry ​[145]. The use of CNT-embedded hydrogel sheets in engineering cardiac constructs and bioactuators was reported ​[146]. Functional cardiac patches were prepared by seeding neonatal rat cardiomyocytes onto CNT-gelatinmethacrylate (GelMA) hydrogels. The resulting cardiac constructs showed excellent mechanical integrity and advanced electrophysiological functions: myocardial tissues cultured on 50 ​μm thick CNT-GelMA showed three times higher spontaneous synchronous beating rates and 85% lower excitation threshold, compared to those cultured on pristine GelMA hydrogels. Protein/peptide-nanocarbon systems indisputably attract strong interest owing to their complementary properties for biological applications, although they are laboriously difficult to design and control ​[147,148].

## Conclusions

Self-assembled nanostructures forming an extended π electron-rich system ​provide an opportunity to develop new semiconductor materials for a variety of applications ranging from organic electronics to bioelectronics ​[7,149]. Electroactive and photoactive self-assembled peptide-based nanostructures were developed as organic electronic materials. These bioinspired materials were designed with aromatic residues/moieties for optical, conductive, ferroelectric, and electrochemical features. Supramolecular polymerization of self-assembling units was achieved in solution as well as from vaporous phase, thus demonstrating versatility of peptide-based molecules in the development of novel materials with unique electronic properties. Electroactive peptide-based supramolecular materials can find applications in regenerative medicine and bioelectronics at the interface of biological tissues.

The article "Electroactive peptide-based supramolecular polymers" was retracted in 2022. Reason: plagiarism.

## Declaration of competing interest

The authors declare that they have no known competing financial interests or personal relationships that could have appeared to influence the work reported in this paper.
